The article "Six2 promotes non–small cell lung cancer cell stemness via transcriptionally and epigenetically regulating E‐cadherin" was retracted in 2024. Reasons: plagiarized images; overlap with other authors' work; original data or images not available; unreliable results or conclusions.

# Six2 promotes non–small cell lung cancer cell stemness via transcriptionally and epigenetically regulating E‐cadherin

**DOI:** 10.1111/cpr.12617

**Published:** 2019-04-22

**Authors:** Huaying Hou, Xiaoming Yu, Ping Cong, Yong Zhou, Ying Xu, Yuhua Jiang

**Affiliations:** ^1^ Cancer Prevention Center The Second Hospital of Shandong University Tianqiao District, Jinan China

**Keywords:** cisplatin, E‐cadherin, non–small cell lung cancer, six2, stemness

## Abstract

**Objectives:**

The roles and related mechanisms of six2 in regulating non–small cell lung cancer (NSCLC) cells progression are unclear. This work aimed to explore the roles of six2 in NSCLC cell stemness.

**Materials and Methods:**

Kaplan‐Meier plotter analysis was used to examine the correlation between six2 expression and the survival of NSCLC patients. Quantitative reverse transcription PCR and Western blot were performed to detect six2 expression in clinical samples. Moreover, transwell migration, tumour spheroid formation and in vivo tumour formation assays were used to examine the effects of six2 on NSCLC cell progression. Additionally, methylation analysis was carried out to measure E‐cadherin methylation level in different cells. Finally, cell viability assay was performed to explore the effects of six2 on chemotherapeutic sensitivity of NSCLC cells.

**Results:**

Lung cancer patients with a higher six2 expression level displayed a shorter overall survival. Six2 expression was higher in lung cancer tissues than in normal adjacent tissues. Additionally, six2 knockdown suppressed NSCLC cell stemness. Mechanistically, six2 overexpression inhibited epithelial marker E‐cadherin expression via stimulating its promoter methylation. And E‐cadherin knockdown rescued six2 knockdown‐induced decrease of NSCLC cancer cell stemness. Notably, six2 knockdown enhanced cisplatin sensitivity in parental NSCLC cells and attenuated cisplatin resistance in cisplatin‐resistant NSCLC cells.

**Conclusions:**

Our results suggest that six2 facilitates NSCLC cell stemness and attenuates chemotherapeutic sensitivity via suppressing E‐cadherin expression.

## 1 INTRODUCTION

Lung cancer is one of the malignant tumours with the highest morbidity and mortality, especially non–small cell lung cancer (NSCLC).^1^ Although surgery, chemotherapy, radiotherapy, molecular targeted therapy and immunotherapy have greatly improved NSCLC patients survival and prognosis, most of patients do not respond to immunotherapy, and tumour recurrence and drug resistance are the main obstacle in clinic.^2^ Thus, identification of and research on novel biomolecules and signalling involved in NSCLC tumorigenesis and progression are of great importance.

The article "Six2 promotes non–small cell lung cancer cell stemness via transcriptionally and epigenetically regulating E‐cadherin" was retracted in 2024. Reasons: plagiarized images; overlap with other authors' work; original data or images not available; unreliable results or conclusions.

The theory of cancer stem cells (CSCs) believes that tumour progression is contributed by CSCs or cells with stemness which hold the ability of self‐renewal and differentiation.^3^ In NSCLC progression, cells with stemness contribute to tumour recurrence, metastasis and chemoresistance,^4^ for example, IL22 promotes lung cancer progression via protection of lung cancer cell stemness properties.^5^ Targeting USP22 attenuates tumorigenicity and enhances chemotherapeutic sensitivity through downregulating lung cancer cell stemness.^6^ And miR‐124a could enhance gefitinib sensitivity of lung cancer cells via attenuating stemness.^7^ Although various studies have elucidated the mechanisms contributing to lung cancer cell stemness, the regulatory mechanisms of lung cancer cell stemness are still confused. Additionally, novel biomolecules and signalling involved in lung cancer stemness must be further explored.

Transcriptional factor six2, a mesenchymal‐epithelial transition, has been shown to promote metanephric mesenchyme cell proliferation and restrain cell apoptosis during kidney development.^8^ And six2 deficiency contributes to mesenchyme progenitors deletion, differentiation dysregulation and severe kidney hypoplasia.^9^ Additionally, six2 could define and regulate a multipotent self‐renewing nephron progenitor population throughout mammalian kidney development.^8^ A previous study has shown that six2 promotes breast cancer metastasis.^10^ Notably, cancer cell stemness could result in cells metastasis.^11^ And since gene expression programmes and cellular processes that are utilized in embryogenesis are often reinstated in tumours,^10^, ^12^ and epithelial‐mesenchymal transition (EMT) process could confer tumour cell stemness,^13^ we deduce that six2 misexpression is involved in lung cancer cell stemness. E‐cadherin, the epithelial marker of EMT, acts as a tumour suppressor in tumour metastasis and stemness^14^; however, the mechanisms by which E‐cadherin is regulated in NSCLC are still unclear.

In the present study, we found that six2 expression was significantly increased in NSCLC tissues and KM plotter analysis showed that six2 expression was negatively correlated with the survival of lung cancer patients. Notably, six2 expression was significantly increased in cisplatin‐resistant NSCLC cells, which displayed a stronger stemness compared with the parental cells. Further in vitro and in vivo experiments indicate that six2 conferred NSCLC cell stemness, and cisplatin resistance. Mechanistically, we found that six2 overexpression inhibited epithelial marker E‐cadherin expression via stimulating its promoter methylation, and E‐cadherin knockdown rescued the inhibition of six2 knockdown on NSCLC cell stemness. Therefore, our results demonstrate that six2 promotes NSCLC cell stemness and chemoresistance via transcriptional and epigenetic control of E‐cadherin expression.

The article "Six2 promotes non–small cell lung cancer cell stemness via transcriptionally and epigenetically regulating E‐cadherin" was retracted in 2024. Reasons: plagiarized images; overlap with other authors' work; original data or images not available; unreliable results or conclusions.

## 2 MATERIAL AND METHODS

### 2.1 Clinical samples and cell culture

Total 61 pairs of NSCLC and normal adjacent clinical samples were obtained from the Second Hospital of Shandong University from March 2016 to January 2018. The Ethics Committees of the Second Hospital of Shandong University has approved this research, and written informed consent from all patients was acquired before using. Human NSCLC cell line A549 and NCI‐H1299 cells, and HEK293T cells and normal lung epithelial cell line BEAS‐2B were purchased from the Chinese Academy of Sciences Cell Bank (Shanghai), and cisplatin‐resistant NSCLC cells (A549‐DDP) were purchased from KeyGen BioTECH (Nanjing). All of the NSCLC and BEAS‐2B cell lines were cultured in 1640 medium (Gibco) containing 10% foetal bovine serum (FBS; Life Technologies) at 37°C with 5% CO_2_. HEK293T cells were cultured in DMEM medium (Gibco), and the other conditions were the same with NSCLC cell lines. Cisplatin (Cat # S1166) was purchased from Selleck.cn.

### 2.2 Lentivirus vectors and stable expression cell lines construction

Six2 coding sequences were inserted into pLVX‐IRES‐ZsGreen1, named as Lenti‐six2. shRNAs against six2, E‐cadherin and a scramble non‐targeting shRNA were purchased from Santa Cruz. The shRNA sequences were inserted into pLKO.1, named as Lenti‐six2‐shRNA, Lenti‐E‐cadherin‐shRNA and control, respectively. Lentivirus was packaged in HEK293T cells via co‐transfecting above‐mentioned constructs, pCMV‐dR8.2 and pMD2.G constructs by Lip2000 (Invitrogen). 48 and 72 hours later, the supernatants were collected and ultrafiltrated. The virus supernatants were added to A549, NCI‐H1299 and A549‐DDP cells with 2 µg/mL polybrene, and followed by screening with puromycin (1.5 µg/mL for A549 and NCI‐H1299 cells, and 2 µg/mL for A549‐DDP cells), the stable six2 knockdown cells were named as A549‐six2‐shRNA, H1299‐six2‐shRNA and A549‐DDP‐six2‐shRNA, respectively.

### 2.3 Cell spheroid formation assay

A total of 2000 single cells were seeded into the 24‐well ultra‐low attachment plate (Corning) in serum‐free DMEM/F12 (Invitrogen), supplemented with B27 (1:50, Invitrogen), 20 ng/mL EGF (PeproTech), 20 ng/mL bFGF (Invitrogen), 100 U/mL penicillin and 100 mg/mL streptomycin and 20% methylcellulose (Sigma). Non‐adherent spheroid number and size were detected and photographed using a microscope fitted with a ruler.

### 2.4 Quantitative real‐time PCR

Quantitative real‐time PCR (qRT‐PCR) was used to examine the relative expression of mRNA. Briefly, total RNA was extracted using Trizol reagent (KeyGEN BioTECH). Then, cDNA was synthesized using reverse transcription PCR kit (KeyGEN BioTECH) following the standard protocols. Afterwards, mRNA expression was examined using real‐time PCR Master Mix (SYBR Green) (KeyGEN BioTECH) and determined on an ABI Prism 7500 Detection System (Applied Biosystems, Inc). Relative mRNA expression was calculated with $2^{-\Delta \Delta {\text{C}}_{t}}$ method. GAPDH served as an internal control for mRNA expression.

The article "Six2 promotes non–small cell lung cancer cell stemness via transcriptionally and epigenetically regulating E‐cadherin" was retracted in 2024. Reasons: plagiarized images; overlap with other authors' work; original data or images not available; unreliable results or conclusions.

### 2.5 DNA methylation analysis

MethPrimer (http://www.urogene.org/cgi-bin/methprimer/methprimer.cgi) was used to analyse the CpG islands on E‐cadherin promoter. Genomic DNA was extracted using EasyPure Genomic DNA Kit (TRANSGEN BIOTECH). Genomic DNA was treated with sodium bisulphite using the CpGenome DNA Modification Kit (Serologicals Corp) following the manufacturer's recommendation. PCR primers were designed to expand E‐cadherin promoter sequences with nuclear CpG island region or not. qRT‐PCR was performed to measure the E‐cadherin promoter level with nuclear CpG island region.

### 2.6 Western blot

Protein was extracted using protein extraction kit (KeyGEN BioTECH), and protein concentration was determined by BCA Protein Assay Kit (KeyGEN BioTECH). 30 μg of protein was separated by SDS‐PAGE and transferred onto PVGF membranes, which were followed by incubating with 5% non‐fat milk for 1.5 hours at room temperature. Afterwards, membranes were incubated with the primary antibodies against six2 (ab132611), ALDH1 (ab23375), Nanog (ab21624), cleaved caspase 3 (ab2302), caspase 3 (ab13847), cleaved PARP (ab32064), PARP (ab74290), which were purchased from Abcam. Primary antibody against β‐actin (cat # AF0003) was purchased from Beyotime. After incubating with primary antibodies, blots were washed and incubated with a secondary peroxidase‐conjugated antibody (KeyGEN BioTECH), and chemiluminescence was detected using an enhanced chemiluminescence kit (ThermoFisher Scientific) followed by exposure in Tanon 5200 (Tanon).

### 2.7 Kaplan‐Meier plotter analysis

Kaplan‐Meier (KM) plotter analysis (http://kmplot.com) was used to analyse the correlation between transcript expression and, overall survival (OS) and first progression of lung cancer patients, in which patients were split by the median expression of six2, and 1928 lung cancer patients were included with all subtypes for OS analysis, and 982 lung cancer patients for first progression analysis.

### 2.8 Cell viability assay

Cells were digested, re‐suspended and seeded into 96‐well plates, followed by the treatment of cisplatin, after 24, 48 and 72 hours, cell viability was examined by CCK8 assay kit (Cat # HY‐K0301; MedChemExpress) following the manufacturer's recommendation.

The article "Six2 promotes non–small cell lung cancer cell stemness via transcriptionally and epigenetically regulating E‐cadherin" was retracted in 2024. Reasons: plagiarized images; overlap with other authors' work; original data or images not available; unreliable results or conclusions.

### 2.9 ALDH1 activity assay

ALDH1 activity was assayed by ALDEFLUOR™ Kit (Cat # KA3742, Stemcell Technologies) following the standard procedure.

### 2.10 Transwell migration analysis

The detailed procedure was referred to the previous work.^15^

### 2.11 In vivo tumorigenic assay

Four‐ to six‐week male athymic BALB/c nude mice were purchased from Model Animal Research Center of Nanjing University, were housed and fed in standard pathogen‐free conditions. For tumour‐limiting dilution assays, NSCLC cells or cell spheroids were mixed 1:1 with Matrigel matrix (BD Biosciences) and subcutaneously implanted in the mice. On day 8, all mice were killed, and tumour tissues were collected and weighed. All animal studies were approved by the Institutional Animal Care and Use Committee of the Second Hospital of Shandong University.

### 2.12 Statistical analysis

Data were presented as the mean ± standard deviation (*SD*). The differences between the groups were analysed using ANOVA with the Tukey‐Kramer post‐test, and *P* < 0.05 was considered statistically significant.

## 3 RESULTS

### 3.1 Six2 expression is significantly upregulated in NSCLC tissues and negatively correlated with the OS of lung cancer patients

We firstly detected six2 expression in NSCLC and normal adjacent tissues and found that six2 expression was significantly increased in NSCLC tissues via qRT‐PCR (Figure 1A), Western blot (Figure 1B) and immunohistochemistry (Figure 1C) assays. Notably, the KM plotter analysis showed that six2 expression was negatively correlated with the first progression and OS of lung cancer patients (Figure 1D,E). Additionally, six2 expression was determined in NSCLC and normal lung epithelial cells. As shown in Figure 1F,G, six2 expression was significantly upregulated in NSCLC A549 and H1299 cells compared with that in normal lung epithelial cell line BEAS‐2B cells. These results suggest that six2 might contribute to NSCLC progression.

**Figure 1:** Six2 expression is significantly upregulated in NSCLC tissues and negatively correlated with the OS of lung cancer patients. A, Six2 mRNA was detected in NSCLC and normal tissues via qRT‐PCR assay. B, C, Six2 protein level was examined in NSCLC and normal tissues via Western blot and immunohistochemistry assays. D, E, The correlation between six2 expression and the first progression, and OS of lung cancer patients was analysed via KM plotter assay. F, G, Six2 mRNA (F) and protein (G) level were determined in NSCLC cells and normal lung epithelial cells. Data were presented as mean ± *SD*; *P < 0.05, **P < 0.01 vs normal tissues or BEAS‐2B

The article "Six2 promotes non–small cell lung cancer cell stemness via transcriptionally and epigenetically regulating E‐cadherin" was retracted in 2024. Reasons: plagiarized images; overlap with other authors' work; original data or images not available; unreliable results or conclusions.

### 3.2 Six2 expression is increased in NSCLC spheroids, which display a stronger stemness relative to parental cells

As tumour cell stemness contributes to tumour metastasis and drug resistance,^11^ we wondered whether six2 was involved in NSCLC cell stemness and thus metastasis. Since 3D culturing non‐adherent spheroids were confirmed to be enriched with tumour cells with strong stemness, A549 and H1299 cells were cultured in ultra‐low attachment plates with the medium depicted in the section of cell spheroid formation assay, and cell spheroids were observed after 8‐day culture (Figure 2A). Indeed, NSCLC spheroids exhibited a stronger stemness characterized as the increase of tumour stemness marker expression (ALDH1 and Nanog) (Figure 2B,C) and ALDH1 activity (Figure 2D). Importantly, NSCLC spheroids were digested and re‐seeded in ultra‐low attachment plates, and displayed a higher spheroid size and number compared with parental cells (Figure 2E,F). Additionally, the tumour‐initiating ability of NSCLC spheroids was stronger than the parental cells characterized as the increase of tumour size (Figure 2G). Notably, six2 expression was remarkably increased in NSCLC spheroids (Figure 2H). Thus, we speculated that six2 might involve in NSCLC cell stemness.

**Figure 2:** Six2 expression is increased in NSCLC spheroids, which display a stronger stemness relative to parental cells. A, Cell spheroid formation ability was examined in A549 and NCI‐H1299 cells. B, C, Expression of stemness markers (ALDH1 and Nanog) was measured in NSCLC cells spheroids and parental cells via qRT‐PCR (B) and Western blot (C) assays. D, ALDH1 activity was determined in the cells depicted in (B). E, F, The formation ability of second generation of spheroids in NSCLC spheroids and cells was detected characterized as the spheroid number and size. G, Images of tumours harvested when NSCLC spheroids and cells were planted. H, I, Six2 mRNA (H) and protein (I) levels were examined in NSCLC cell spheroids and cells. Data were presented as mean ± *SD*; *P < 0.05, **P < 0.01 vs A549 or NCI‐H1299

### 3.3 Knockdown of six2 attenuated NSCLC cell stemness

Then, we detected whether six2 contributed to NSCLC cell stemness. Since six2 expression was upregulated in NSCLC cells, we constructed six2 stable knockdown NSCLC cells with lentivirus infection, qRT‐PCR and Western blot analysis confirmed the knockdown efficiency of six2 (Figure 3A,B). As expected, six2 knockdown suppressed the expression of stemness markers (ALDH1 and Nanog) (Figure 3C,D) and ALDH1 activity (Figure 3E). Additionally, cell spheroid formation assay showed that six2 knockdown attenuated the spheroid formation characterized as the decrease of spheroid size and number (Figure 3F,G). We further compared the capacity of NSCLC cells with or without six2 knockdown to seed tumours at limiting dilutions. Notably, the tumour‐seeding ability of six2 knockdown NSCLC cells was significantly decreased at the density of 1 × 10^5^ and 1 × 10^4^ cells, respectively, characterized as the decrease of tumour size and number (Figure 3H).

The article "Six2 promotes non–small cell lung cancer cell stemness via transcriptionally and epigenetically regulating E‐cadherin" was retracted in 2024. Reasons: plagiarized images; overlap with other authors' work; original data or images not available; unreliable results or conclusions.

**Figure 3:** Knockdown of six2 attenuated NSCLC cell stemness. A, B, Knockdown efficiency of six2 was measured in NSCLC cells with six2 stable knockdown or not via qRT‐PCR (A) and Western blot (B) assay. C, D, Expression of stemness markers (ALDH1 and Nanog) was detected in the cells depicted in (A) via qRT‐PCR and Western blot assay. E, ALDH1 activity was examined in cells depicted in (A). F, G, Spheroid size (F) and number (G) of NSCLC cells with or without six2 knockdown were determined. H, Images of tumours harvested when serially diluted NSCLC cells with or without six2 knockdown were planted. Data were presented as mean ± *SD*; *P < 0.05, **P < 0.01 vs A549 or NCI‐H1299

### 3.4 Knockdown of six2 attenuated NSCLC cell migration

Since tumour cell stemness could lead to cell metastasis, we continue exploring the effects of six2 knockdown on NSCLC cell migration ability. Transwell migration assay showed that six2 knockdown decreased the migration ability of NSCLC cells (Figure 4A,B). Additionally, six2 knockdown attenuated the EMT process in NSCLC cells characterized as the decrease of mesenchymal marker (Vimentin) expression and increase of epithelial marker (E‐cadherin) expression (Figure 4C,D). Therefore, our results demonstrate that six2 knockdown decreased NSCLC cell stemness and thus migration ability.

**Figure 4:** Knockdown of six2 attenuated NSCLC cells migration. A, B, Migration ability was examined and quantified in NSCLC cells with six2 knockdown or not. C, D, The expression of EMT markers (E‐cadherin and Vimentin) was detected in NSCLC cells with or without six2 knockdown. Data were presented as mean ± *SD*; *P < 0.05, **P < 0.01 vs A549 or NCI‐H1299

### 3.5 Six2 overexpression inhibited epithelial marker E‐cadherin expression via stimulating its promoter methylation

The previous study has indicated that the decrease of E‐cadherin expression is resulted by DNA methylation in human cancers.^16^ We asked whether E‐cadherin promoter methylation was the mechanism contributing to six2‐mediated downregulation of E‐cadherin, NSCLC cells with six2 overexpression were treated with the methyltransferase inhibitor 5 μmol/L decitabine, and E‐cadherin expression was partially restored, while no further increase in E‐cadherin expression was observed in control cells (Figure 5A,B). Methylation analysis of the E‐cadherin promoter revealed that cells with six2 overexpression had a significant increase in E‐cadherin CpG island methylation (Figure 5C). Additionally, NSCLC cells expressing a high level of six2 and a low level of E‐cadherin were followed by a high level of E‐cadherin promoter methylation, while normal lung epithelial BEAS‐2B cells expressing a low level of six2 and a high level of E‐cadherin had correspondingly a low level of E‐cadherin promoter methylation (Figure 5D). Notably, the expression of six2 and E‐cadherin was negatively correlated in NSCLC tissues (Figure 5E). Taken together, our results suggest that six2 could inhibit E‐cadherin expression via altering the methylation status of its promoter.

The article "Six2 promotes non–small cell lung cancer cell stemness via transcriptionally and epigenetically regulating E‐cadherin" was retracted in 2024. Reasons: plagiarized images; overlap with other authors' work; original data or images not available; unreliable results or conclusions.

**Figure 5:** Six2 overexpression inhibited epithelial marker E‐cadherin expression via stimulating its promoter methylation. A, B, E‐cadherin mRNA (A) and protein (B) levels were detected in NSCLC cells with or without six2 overexpression plus DNA methylation inhibitor (Decitabine) treatment or not. C, Genomic DNA from HCC cells with or without six2 overexpression was collected, and E‐cadherin promoter CpG methylation status was examined using EpiTech Methyl II PCR primer assay for the E‐cadherin promoter. D, The methylated level of E‐cadherin was measured in A549, NCI‐H1299 and BEAS‐2B cells. E, The correlation between six2 and E‐cadherin expression was analysed in NSCLC tissues. Data were presented as mean ± *SD*; *P < 0.05, **P < 0.01 vs A549 or H1299.

### 3.6 Six2 promotes NSCLC cell stemness and migration partly dependent on E‐cadherin expression

We further investigated whether the inhibition of six2 knockdown on NSCLC cell stemness and migration was dependent on E‐cadherin expression. E‐cadherin expression was knocked down in NSCLC cells with six2 knockdown via lentivirus infection, qRT‐PCR and Western blot confirmed the knockdown efficiency and knockdown of E‐cadherin rescued the inhibition of six2 knockdown on the expression of stemness markers (ALDH1 and Nanog) (Figure 6A‐D). Further ALDH1 activity assay showed that E‐cadherin knockdown attenuated the inhibition of six2 knockdown on ALDH1 activity (Figure 6E). Additionally, the decrease of spheroid formation ability induced by six2 knockdown was rescued by E‐cadherin knockdown (Figure 6F,G). Moreover, E‐cadherin knockdown attenuated the inhibition of six2 knockdown on NSCLC cell migration (Figure 6H). Notably, the tumour‐seeding ability of six2 knockdown NSCLC cells was significantly rescued by E‐cadherin knockdown at the density of 1 × 10^4 ^cells (Figure 6I).

The article "Six2 promotes non–small cell lung cancer cell stemness via transcriptionally and epigenetically regulating E‐cadherin" was retracted in 2024. Reasons: plagiarized images; overlap with other authors' work; original data or images not available; unreliable results or conclusions.

**Figure 6:** Six2 promotes NSCLC cell stemness and migration partly dependent on E‐cadherin expression. A, B, The mRNA levels of stemness markers (ALDH1 and Nanog) were detected in NSCLC cells with six2 knockdown plus E‐cadherin knockdown or not. C, D, The protein levels of stemness markers (ALDH1 and Nanog) and E‐cadherin were examined in NSCLC cells depicted in (A). E, ALDH1 activity was measured in the cells depicted in (A). F, G, Spheroids size and number was detected in the cells depicted in (A). H, Migration ability was determined in the cells depicted in (A). I, Images of tumours harvested when NSCLC cells depicted in (A) at the density of 1 × 10^4 ^cells were planted. Data were presented as mean ± *SD*; *P < 0.05, **P < 0.01 vs A549 or NCI‐H1299

### 3.7 Six2 Knockdown of attenuated cisplatin resistance of A549‐DDP cells

As tumour cell stemness contributed to drug resistance, we further explored whether six2 knockdown could attenuate chemoresistance of A549‐DDP cells. Firstly, we compared the stemness of A549 and A549‐DDP cells and found that A549‐DDP cells indeed displayed a higher stemness relative to A549 cells, characterized as the increased expression of stemness markers (ALDH1 and Nanog) (Figure 7A,B), increase of ALDH1 activity (Figure 7C) and spheroid formation ability (Figure 7D,E). Additionally, both NSCLC cell spheroids and A549‐DDP cells displayed a higher expression of drug resistance genes (ABCG2 and MDR1) compared with that in parental cells (Figure 7F,G). Notably, six2 expression was significantly increased in A549‐DDP cells (Figure 7H). Then, we constructed A549‐DDP cells with six2 stable knockdown and showed that six2 knockdown attenuated A549‐DDP cell stemness (Figure 8). Further cell viability and apoptosis analysis indicated that six2 knockdown attenuated the cisplatin resistance of A549‐DDP cells (Figure 7I,J). Western blot analysis on apoptosis executor (cleaved caspase 3 and cleaved PARP) expression acquired the consistent results (Figure 7K). Importantly, six2 knockdown enhanced cisplatin sensitivity in parental A549 cells (Figure 9). Therefore, our results demonstrate that six2 knockdown could re‐sensitize A549‐DDP cells to cisplatin and enhance cisplatin sensitivity in A549 cells via attenuating cell stemness.

**Figure 7:** Knockdown of six2 attenuated cisplatin resistance of A549‐DDP cells. A, B, Expression of stemness markers (ALDH1 and Nanog) was detected in A549 and A549‐DDP cells via qRT‐PCR (A) and Western blot (B) assay. C, ALDH1 activity was measured in A549 and A549‐DDP cells. D, E, Spheroid size and number were examined in A549 and A549‐DDP cells. F, G, Expression of drug resistance genes (ABCG2 and MDR1) was determined in A549 cells, A549 spheroids and A549‐DDP cells. H, Six2 expression was detected in A549 and A549‐DDP cells. I, J, A549‐DDP cells with or without six2 knockdown were treated with cisplatin, and followed by cell viability (I) and cell apoptosis (J) assay. K, Expression of apoptosis executors (cleaved caspase 3 and cleaved PARP) was examined in the cells depicted in (I). Data were presented as mean ± *SD*; *P < 0.05, **P < 0.01 vs A549‐DDP or A549

**Figure 8:** Knockdown of six2 attenuates A549‐DDP cell stemness. A, B, Expression of stemness markers (ALDH1 and Nanog) was determined in A549‐DDP cells with or without six2 knockdown. C, ALDH1 activity was detected in A549‐DDP cells with or without six2 knockdown. D, E, Spheroid size and number were measured in A549‐DDP cells with or without six2 knockdown. Data were presented as mean ± *SD*; *P < 0.05, **P < 0.01 vs A549

**Figure 9:** Knockdown of six2 enhances cisplatin sensitivity of A549 cells. A, B, A549 cells with or without six2 knockdown were treated with cisplatin, and followed by cell viability (A) and apoptosis (B) assay. C, Expression of apoptosis executors (cleaved caspase 3 and cleaved PARP) was examined in the cells depicted in (A). Data were presented as mean ± *SD*; **P < 0.01 vs A549

The article "Six2 promotes non–small cell lung cancer cell stemness via transcriptionally and epigenetically regulating E‐cadherin" was retracted in 2024. Reasons: plagiarized images; overlap with other authors' work; original data or images not available; unreliable results or conclusions.

## 4 DISCUSSION

Although a large number of evidence have elucidated the molecular signalling contributing to tumour heterogeneity,^17^, ^18^ the detailed mechanisms contributing to the tumour heterogeneity and drug resistance of lung cancer are still unclear. Studies have suggested that abnormal activation of signalling pathways associated with embryonic development or division and differentiation is correlated with tumour recurrence and metastasis, like Notch signalling plays an important role in regulating embryo development, and has been shown to be involved in promoting tumour stem cell generation and maintenance.^19^, ^20^ And Hedgehog pathway plays an important role in embryonic development, and in the repair and regeneration of adult tissue. Meanwhile, the abnormal activation of Hedgehog pathway is linked with brain, skin, gastrointestinal tract and pancreas cancers.^21^

As transcriptional factor six2 could define and regulate a multipotent self‐renewing nephron progenitor population throughout mammalian kidney development,^8^ we believe that six2 plays important roles in tumour progression, especially in NSCLC which displays high morbidity and mortality. Previous studies have shown that six2 is required for DDX3‐mediated tumour aggressiveness and cetuximab resistance in KRAS‐wild‐type colorectal cancer,^22^ has been confirmed to facilitate breast cancer metastasis.^10^ Recent study has demonstrated that six2 is negatively correlated with good prognosis and decreases 5‐FU sensitivity in hepatocellular carcinoma cells via regulating cell stemness.^23^ However, the roles and related mechanism in NSCLC progression are still unclear. Here, we found that six2 expression was significantly increased in NSCLC tissues and cells, and cisplatin‐resistant NSCLC cells. Functional experiments showed that knockdown of six2 attenuated NSCLC cell stemness and migration, re‐sensitized cisplatin‐resistant cells to cisplatin and enhance cisplatin sensitivity in NSCLC cells. Notably, our results were consistent with the recent work showing that six2 promoting the stemness of breast cancer cells.^24^, ^25^ To the best of our knowledge, this is the first study showing the roles of six2 in NSCLC migration and stemness.

The article "Six2 promotes non–small cell lung cancer cell stemness via transcriptionally and epigenetically regulating E‐cadherin" was retracted in 2024. Reasons: plagiarized images; overlap with other authors' work; original data or images not available; unreliable results or conclusions.

Notably, our results indicated that NSCLC cells expressing a high level of six2 and a low level of E‐cadherin were followed by a high level of E‐cadherin promoter methylation. In contrast, normal lung epithelial BEAS‐2B cells expressing a low level of six2 and a high level of E‐cadherin had correspondingly a low level of E‐cadherin promoter methylation, and these effects were consistent with the previous work showing that the decrease of E‐cadherin expression is resulted by DNA methylation in human cancers.^16^ Importantly, we found that six2 expression was negatively correlated with E‐cadherin expression in NSCLC tissues, and six2 promoted E‐cadherin methylation. Although the effect of six2 on E‐cadherin methylation has been confirmed in breast cancer,^10^ our work further confirmed the interaction between six2 and E‐cadherin in NSCLC. Future works could explore whether the interaction between six2 and E‐cadherin was a common phenomenon in other tumours. Since E‐cadherin knockdown could not reverse the inhibition of six2 knockdown on NSCLC cell stemness and migration, we speculated that the other pathways might be involved in the regulation of six2 on E‐cadherin expression, such as miRNAs are involved in the regulation of six2 on E‐cadherin expression in breast cancer,^10^ which is also needed to further validation.

Many works have been exploring methods regulating lung cancer cell stemness and thus attenuating drug resistance. For example, Niu et al have shown that low molecular weight heparin could attenuate cisplatin resistance of A549‐DDP cells via downregulating cell stemness.^26^ Yeh et al^27^ have indicated that trifluoperazine could effectively decrease gefitinib or cisplatin resistance of lung cancer cells via targeting lung cancer cells with strong stemness. These works suggest that it is an effective way to treat lung cancer via attenuating cell stemness. This work reveals that six2 could facilitate NSCLC stemness and attenuate cisplatin sensitivity. Our results demonstrate that downregulation of six2 could be a potential predictive marker as well as novel therapeutic target in future NSCLC treatment.
